# Auraptene-induced cytotoxicity mechanisms in human malignant glioblastoma (U87) cells: role of reactive oxygen species (ROS)

This article has been retracted.

**DOI:** 10.17179/excli2019-1136

**Published:** 2019-07-30

**Authors:** Amir R. Afshari, Mohammad Jalili-Nik, Mohammad Soukhtanloo, Ahmad Ghorbani, Hamid R. Sadeghnia, Hamid Mollazadeh, Mostafa Karimi Roshan, Farzad Rahmani, Hamed Sabri, Mohammad Mahdi Vahedi, Seyed Hadi Mousavi

**Affiliations:** 1 Department of Physiology and Pharmacology, School of Medicine, North Khorasan University of Medical Sciences, Bojnurd, Iran; 2 Department of Pharmacology, Faculty of Medicine, Mashhad University of Medical Sciences, Mashhad, Iran; 3 Department of Clinical Biochemistry, Faculty of Medicine, Mashhad University of Medical Sciences, Mashhad, Iran; 4 Pharmacological Research Center of Medicinal Plants, Mashhad University of Medical Sciences, Mashhad, Iran; 5 Department of Pharmacology, School of Medicine, Zahedan University of Medical Sciences, Zahedan, Iran; 6 Health Promotion Research Center, Zahedan University of Medical Sciences, Zahedan, Iran; 7 Medical Toxicology Research Center, Mashhad University of Medical Sciences, Mashhad, Iran

**Keywords:** glioblastoma multiforme, auraptene, ROS, apoptosis

## Abstract

Glioblastoma multiforme (GBM), like the devastating type of astrocytic tumors, is one of the most challenging cancers to treat owing to its aggressive nature. Auraptene, as a prenyloxy coumarin from citrus species, represents antioxidant and antitumor activities; however, the underlying antitumor mechanisms of auraptene against GBM remain unclear. The present study aimed to evaluate the cytotoxic and apoptogenic effects of auraptene, as a promising natural product, and the possible signaling pathways affected in human malignant GBM (U87) cells. Reactive oxygen species (ROS) production significantly decreased in the first 2, and 6 hours after treatment with auraptene however, ROS levels increased in other incubation times (8 and 24 hours), dramatically. N-acetyl-cysteine (NAC) markedly attenuated auraptene-induced ROS production, and consequently reversed auraptene-induced cytotoxicity in 8 and 24 hours after treatment, as well. Induction of apoptosis occurred in the first 24- and 48-hours concentration-dependently. The qRT-PCR showed an up-regulation in p21, CXCL3, and a down-regulation in Cyclin D1 genes expression. Western blot analysis confirmed the up-regulation of the Bax/Bcl-2 ratio protein levels concentration-dependently. Hence, this study collectively revealed that the increase in ROS level is at least one of the mechanisms associated with auraptene-induced GBM cell toxicity as well as the induction of apoptosis through Bax/Bcl-2 modulation and genes expression involved that contribute to the cytotoxicity of auraptene in U87 cells. So, auraptene might be utilized as a potential novel anti-GBM agent after further studies.

## Introduction

Glioblastoma multiforme (GBM) is the deadliest primary astrocytic tumor with high cell proliferation and one-year survival rate. Indeed, even the most utilized conventional GBM therapy, including surgical resection, local irradiation, and chemotherapy may only increase an average of two-months survival of patients (Yang et al., 2018[52]). So, a novel therapeutic approach to treat this malignant disease is crucial.

Auraptene (Figure 1(Fig. 1)), belongs to the Rutaceae and Apiaceae plant families, has been recognized to possess promising various pharmacological properties (Murakami et al., 1997[27], 2000[28][29]; Tanaka et al., 1997[45], 1998[44], 2000[46]; Soltani et al., 2010[40]; Afshari et al., 2019[3]). Although, the antitumor effects of auraptene have been shown recently in various human cancer cells, such as colon, liver, prostate, breast, and skin tumors (Tanaka et al., 1998[44], 2010[43]), the underlying cytotoxic and apoptogenic mechanisms of auraptene in GBM cancer is not fully comprehended to date.

Disruptions in reactive oxygen species (ROS) and defects in apoptotic signaling (Bax/Bcl-2 deregulation) are the primary mechanisms of GBM pathogenesis (Wang et al., 2017[50][51]). Lately, a developing interest has been found to examine the role of ROS during apoptosis induction in different cancer cell lines, including GBM. Various examinations have shown that specific anticancer agents (e.g., doxorubicin, epirubicin, and daunomycin) prompt apoptosis in part with the generation of ROS and the disturbance of redox homeostasis (Long et al., 2007[22]).

According to our knowledge, there are no reports regarding the cytotoxic impacts of auraptene with a focus on ROS production in U87 cells. Hence, the current examination was designed to evaluate the cytotoxic and apoptogenic impacts of auraptene concentrating on ROS production using U87 cells *in vitro*. 

## Materials and Methods

### Cell line and reagents

Auraptene and N-acetyl-cysteine (NAC) were purchased from Cayman Chemical (Michigan, MI, USA). The human malignant GBM (U87) cell line was obtained from the National Cell Bank of Iran (NCBI), Pasteur Institute (Tehran, Iran). The Dichloro-dihydro-fluorescein diacetate (DCFDA)/ H2DCFDA- cellular ROS detection assay kit was obtained from Abcam (Cambridge, United Kingdom). Annexin V-FITC early apoptosis assay kit and antibodies against Bax, Bcl-2, and β-actin were prepared from Cell Signaling Technology (Beverly, MA, USA). Dimethyl sulfoxide (DMSO), gelatin, trypsin-EDTA, and penicillin-streptomycin were provided from Sigma-Aldrich (St. Louis, MO, USA). The bicinchoninic acid (BCA), protein assay kit, was produced by Pierce Co. (Pierce, Rockford, IL, USA). Fetal bovine serum (FBS) and High Glucose-Dulbecco's Modified Eagle's medium (DMEM) were obtained from Gibco (Grand Island, NY, USA). 

### Cell culture and treatment

The U87 cells were kept in an incubator at 37 °C. The cells were cultured in a high glucose DMEM (4.5 g/L) supplemented with 10 % v/v FBS, and 100 unit/mL of penicillin-streptomycin, and the media were changed twice a week. The cells were cultured overnight and then treated with 100 and 400 μg/ mL of auraptene. All the treatments were triplicated. 

### Measurement of ROS levels

This method was performed and analyzed by the DCFDA/H2DCFDA - cellular ROS detection assay kit according to the manufacturer's instructions. The U87 cells (25×10^3^/well) were seeded out overnight in a 96-well dark-sided culture plate. After overnight incubation, the cells were washed with 100 μL of 1X buffer and incubated with 100 μL of H2DCFDA (25 μM) solution for 30-45 minutes in the dark at 37 °C. Then, the cells were rewashed and treated with auraptene (50, 100, 200 µg/mL) or NAC (5 mM) for 2, 6, 8, and 24 hours. The fluorescence was measured at an excitation of 485 nm and emission of 535 nm with the fluorescence plate reader FACScan (Becton Dickinson, San Jose, USA). All treatments were done in triplicate.

### Apoptosis flow cytometry assay 

Early/late apoptosis was detected by the Annexin V/PI staining kit according to the manufacturer's instructions. In brief, after 24 hours of cell incubation (7×10^5^ in a 6-well culture plate) with auraptene (100 and 400 μg/mL), the cells were harvested and washed twice with ice-cold PBS and re-suspended in 200 μL of 1X binding buffer containing Annexin V. Next, 96 µL of cell suspension was transferred to the flow cytometric tube, and then 1 µL of conjugated Annexin V-FITC and PI (12.5 µL) were added to the cells. The cells were incubated for 10 minutes at 0 °C in the dark. After that, the final volume was set at 250 µL with 1X binding buffer containing Annexin V. The number of viable, early apoptotic, late apoptotic, and necrotic cells were quantified immediately by the BD Facscalibur™ flow cytometer (Becton Dickinson, Mountain View, CA, USA). Analysis of the flow cytometry data was done utilizing the software FlowJo^®^ vX.0.7 (Tree Star, Ashland, OR, USA). All treatments were carried out in triplicate.

### Quantitative Real-Time Polymerase Chain Reaction (qRT-PCR)

Total RNA was extracted from the treated U87 cells (7 ×10^5^ cells/well) according to the RNeasy^®^ mini kit protocol (Qiagen GmbH, Hilden, Germany). Next, RNAs were reverse-transcribed utilizing the Prime-Script™ RT reagent kit (TaKaRa Holdings, Inc., Kyoto, Japan). Next, qRT*-*PCR was performed with specific primers for GAPDH, p21, Cyclin D1, and CXCL3 (Table 1(Tab. 1)), which were purchased from Macrogene (Macrogene Co., Seoul, South Korea). The cDNA amplification was done utilizing the Light Cycler 96 RT-PCR system (Roche Applied Science, Pleasanton, CA, USA). The 2^−ΔΔCt^ technique was used to analyze the relative expression of target genes. Gene expression data were normalized to GAPDH. ***‎***

The primer sequences (forward and reverse) are listed in Table 1(Tab. 1).

### Preparation of lysates and Western blot analysis

The 7 × 10^5 ^cells were overnighted and treated with auraptene (100 and 400 μg/mL). After 24 hours of incubation, U87 cells were lysed in RIPA lysis buffer. The lysates were then centrifuged, and the supernatants were maintained at −70 °C before being utilized. The BCA protein assay kit analyzed the proteins concentration. The lysates were separated by 7.5-15% SDS-PAGE and transferred onto a polyvinylidene difluoride (PVDF) membrane (Bio-Rad, HC, USA) utilizing a transfer buffer. After blocking, the membrane was incubated with primary antibodies followed by 2 hours with a secondary antibody. The primary antibodies (1: 1,000) were diluted according to the manufacturer‎'‎s instructions and incubated with the membrane overnight at 4 °C. Then, the horseradish peroxidase-conjugated secondary antibody was added (1: 3,000 dilution) and incubated with the membranes for 1 hour. The detection of each protein was carried out using the SuperSignal^®^ West Femto (Thermo Fisher Scientific, Inc., USA) Western blotting kit according to the manufacturer's instructions. The relative expression was performed using Image J 1.52a software (NIH, Bethesda, Rockville, MD, USA) and then compared to the β-actin protein.

### Statistical analysis

The obtained data were analyzed using the software GraphPad Prism^®^ 7.01 (GraphPad Software, San Diego, CA, USA) and the values were compared using the one-way analysis of variance (ANOVA) followed by the Dunnett test. Furthermore, the study of apoptosis and Western blotting was carried out by FlowJo^®^ vX.0.7 (Tree Star, Ashland, OR, USA) and Image J 1.52a software (NIH, Bethesda, Rockville, MD, USA), respectively. The outcomes are stated as the mean ± standard error. P-values less than 0.05 were considered significant. 

## Results

### The increase of ROS levels in U87 cells by auraptene

To evaluate the role of ROS in auraptene-induced cytotoxicity, we measured the levels of ROS generation using a fluorimeter (Epoch, BioTek^®^ instruments, Inc, USA). As presented in Figure 2A(Fig. 2), the levels of ROS in the cells treated with auraptene showed a significant reduction in the early hours (2 and 6 hours after treatment, p<0.001), and a considerable increase in the 24 hours after treatment (p<0.05). Moreover, ROS level elevation in the 8 hours after treatment by auraptene was not remarkably. 

Blocking the generation of ROS by the treatment of NAC (a ROS scavenger, five mM) not only almost mitigated auraptene-prompted ROS elevation but also reversed the decrease of cell viability at 24 (50, 100 and 200 μg/mL) hours after treatment in U87 cells significantly (Figure 2B(Fig. 2)).

### Auraptene induced apoptosis in U87 cells

To determine apoptosis, we observed apoptotic and necrotic cells at concentrations of 100 and 400 μg/mL as 78.71 % and 95.83 %, respectively, after 24 hours of treatment, as shown in Figure 3A(Fig. 3). Besides, apoptotic and necrotic cells 48 hours after treatment at concentrations of 100 and 400 μg/mL were reported as 76.71 % and 81.47 %, respectively, as shown in Figure 4A(Fig. 4). Furthermore, as shown in Figures 3B(Fig. 3) and 4B(Fig. 4), we summarized the percentage of apoptosis process in each phase. Apoptotic and necrotic index at 24 and 48 hours after treatment was significantly increased in a concentration-dependent manner (Figures 3C(Fig. 3) and 4C(Fig. 4), p<0.001). 

### Impact of auraptene on expression levels of the p21, Cyclin D1, and CXCL3 genes

The results showed that auraptene up-regulated p21 and CXCL3 (P<0.05 and p<0.001) at mRNA level 24 hours after treatment. Also, the expression of Cyclin D1 (P<0.01, and p<0.001, concentration-dependently) gene was mitigated 24 hours after treatment, significantly (Figure 5(Fig. 5)). 

### Impact of auraptene on Bax and Bcl-2 proteins expression

To further illuminate the molecular mechanisms of auraptene affecting U87 cellular apoptosis, Western blotting was used to detect the changes in signaling molecules in U87 cells (Figure 6A(Fig. 6)). 

The analysis of data showed that auraptene significantly affects the function of U87 cells via increasing of Bax (P<0.001), down-regulation of Bcl-2 (100 μg/mL was significant, 400 μg/mL was not significant [P<0.001]) 24 hours after treatment. Also, the Bax/Bcl-2 protein ratio was increased remarkably in both of auraptene concentrations (Figure 6B(Fig. 6)).

## Discussion

GBM, as the most aggressive type of malignant primary brain tumor in humans, is still a serious public health problem because of high morbidity and mortality, regardless of maximal standard treatments (Song et al., 2018[41]; Tang et al., 2017[47]). To date, temozolomide and bevacizumab, have been used as the main chemotherapeutic for treating GBM and ‎preventing its recurrence. Unfortunately, response rates for these drugs are significantly low (Chinot et al., 2014[11]; Hovinga et al., 2019[15]). ‎Given this limited efficacy, finding novel strategies are essential to improve the prognosis of GBM patients. Hence, in the current study, we evaluated the cytotoxic and apoptogenic properties of auraptene, as a ‎potential natural product, against GBM for the first time. 

Natural products have been utilized over the years because of a large number of side effects of chemotherapeutic agents in treating cancer (Asadbeigi et al., 2014[6]; Kaur et al., 2018[18]; Tavakkol-Afshari et al., 2008[48]; Mousavi et al., 2009[24][25]). These agents are usually inexpensive, available, effective, safe, and have fewer side effects (Afshari et al., 2016[4], 2018[2]; Boroushaki et al., 2016[7]; Sadeghnia et al., 2017[34]; Mollazadeh et al., 2017[23]; Shafiee-Nick et al., 2017[36]; Fanoudi et al., 2017[13]). We found that auraptene mechanistically triggers auraptene-induced cytotoxicity through ROS production, up-regulating the Bax/Bcl-2 protein level, and modulating the expression of transcription genes involved in the cell cycle. Various studies have examined the cytotoxic impacts of auraptene in animal models of prostate, liver, breast, intestinal, and skin tumors (Tanaka et al., 2000[46]; Kohno et al., 2006[19]; Jun et al., 2007[16]). In our previous study (Afshari et al., 2019[3]), it was revealed that U87 cell proliferation was influenced by different concentrations of auraptene (0-400 μg/mL), in a time- and concentration-dependent manner (IC_50_ was detected at a concentration of 100 μg/mL). 

ROS, as characterized as oxygen-containing species with reactive properties, assume an essential role in abnormal pathological processes including cancer, particularly brain tumors. Some studies have shown that cancer cells (as compared to normal cells) displayed elevated ROS generation, which was considered to be instigated by an enhanced metabolic activity, mitochondrial dysfunction, and oncogenic incitement (Wang et al., 2017[50][51]). The elevated ROS production in cancer cells not only further promotes genetic instability, stimulates cell proliferation, and formation of drug resistance, but also may give a biochemical basis for therapeutic approaches to kill cancer cells by further increasing ROS generation utilizing pharmacological agents. So, ROS appears to be the critical player in auraptene-induced cell death in cancer (Afshari et al., 2019[3]; Okuyama et al., 2016[31]; Kumar et al., 2016[21]).

In some studies, the effects of antioxidant, anti-inflammation, and apoptosis induction of auraptene were mentioned (Tanaka et al., 2000[46]; Hara et al., 2005[14]; Kostova, 2006[20]). Murakami et al. in their study have shown that auraptene significantly decreased the expression and production of inducible nitric oxide synthase/cyclooxygenase and the release of the tumor necrosis factor (TNF)-α, thereby reducing the production of ROS (Murakami et al., 2000[28][29]; Murakami and Ohigashi, 2006[30]). In the present research, ROS generation mitigated by auraptene in the early hours. However, ROS level at 24 hours after treatment elevated significantly; this impact was plateaued at 24 hours and lower concentration. According to the above, to find out whether this increase was due to cell death induced by auraptene or not, a combination of NAC (5 mM, as an antioxidant agent) plus auraptene in U87 cells were used. It was found that NAC reduced the production of ROS at the last hours of treatment. Also, a significant reduction in the auraptene-induced ROS at 8 and 24 hours was observed. In line with the present outcomes, the production of ROS in inflammation and apoptosis is a crucial role by facilitating the activation of caspase and activating the pathway of NF-κB. Thus, when ROS production is out of control, it can stimulate apoptosis (Su et al., 2005[42]; Dewson and Kluck, 2009[12]; Kagan et al., 2005[17]). Besides, the anti-proliferative impact of auraptene was reversed (at 50 μg/mL concentration of auraptene in 8 hours and a concentration of 100 and 200 in 24 hours) by the treatment of NAC, demonstrating a ROS mediated mechanism of auraptene prompted cytotoxicity in U87 cells. It ought to be noted; auraptene has been recommended to apply potent antioxidant ability in hepatotoxicity (Sahebkar, 2011[35]), which is in contrary to our outcomes in U87 cells. This inconsistency may be clarified by the diverse cell types utilized, or distinct pathophysiologic characters among normal and neoplastic cells, which should be furthermore elucidated. 

Induction of apoptosis is one of the most critical strategies in the prevention and treatment of cancer (Mousavi et al., 2008[26], 2009[24][25]; Tayarani-Najaran et al., 2011[49]; Sharifi et al., 2010[38]; Parsaee et al., 2013[32]), especially astrocytic tumors (Mousavi et al., 2008[26]; Parsaee et al., 2013[32]; Sharma et al., 2017[39]; Piperigkou et al., 2018[33]; Sharifi et al., 2007[37]). Many of the substances used in diets and herbs can have cancer-related effects through their induction of apoptosis (Abu-Darwish and Efferth, 2018[1]). The induction of apoptosis and necrosis in U87 cells by the auraptene was monitored by utilizing fluorescent stains (Annexin V and PI) via flow cytometry. Our outcomes have shown that auraptene effectively induces apoptosis concentration-dependently in U87 cells. The primary cause of death at concentrations of 100 μg/mL (IC_50 _concentration), was apoptosis 24 hours after treatment, and the leading cause of death at 400 μg/mL, was apoptosis and necrosis. In 48 hours after treatment, apoptosis and necrosis were observed, but the main cause of death at a concentration of 100 μg/mL was apoptosis, and the main cause of death at 400 μg/mL was necrosis. In accordance with this study, auraptene had anticancer effects in Jurkat T-cell cells by necrosis and apoptosis after 24 hours (Jun et al., 2007[16]). 

The proportion of Bax to Bcl-2 is a definitive factor in the induction of apoptosis, and the balance between the expression levels of the proteins Bax and Bcl-2 are crucial for cell survival or death. Our previous study was shown that auraptene triggers apoptosis in U87 GBM cells at concentrations of 100 and 400 µg/mL, through the expanded proportion of Bax/Bcl-2 genes expression. 

The present results from the Western blot analysis have shown that a down-regulation of Bcl-2 protein levels and an up-regulation of Bax protein expression was observed 24 hours after treatment. These results suggest that the Bax/Bcl-2 signaling pathway is partly involved in the apoptosis induced by auraptene.

Since auraptene was able to disrupt the cell cycle (discussed in our previous study) and apoptosis induction, the impact of auraptene on the genes involved in the U87 cell cycle was investigated. The results of our study demonstrated that auraptene could reduce the expression of the Cyclin D1 gene at the mRNA level, possibly resulting in a disturbance in the cell cycle. Studies have shown that mutation, amplification, and extreme expression of Cyclin D1, which leads to the progression of the cell cycle, are often observed in a variety of tumors and may lead to tumorigenicity. The expression of Cyclin D1 has up-regulated in breast carcinoma and GBM, leading to increase in the invasion and metastasis (Arato‐Ohshima and Sawa, 1999[5]; Büschges et al., 1999[9]). 

The p21 protein plays a vital role in regulating the cell cycle, proliferation, and stopping cell growth and apoptosis, as well. Studies have revealed that reducing the expression of this protein increases the tumor stage, invasion, and metastasis to the lymph nodes (Chen et al., 1999[10]). The current study showed that the expression of p21 gene expression increased, which was consistent with the results of the cell cycle (discussed in our previous review) and apoptosis.

Also, the present study showed that auraptene at both concentrations (100 and 400 μg/mL) increases the gene expression level of CXCL3 chemokine, which is essential in reducing GBM tumorigenicity. Studies have shown that CXCL3 gene expression controls the migration and adhesion of monocytes and reduces the amount of this chemokine in GBM tumorigenicity. Recently, it has been shown that CXCL3 regulates the cell independently of the migration of progressive cerebellar granular neurons to the cerebellar inner layers during cerebellar morphogenesis. Besides, if the expression of CXCL3 is reduced in brain granulator precursors, this increases the risk of medulloblastoma (Bruyère et al., 2011[8]).

Collectively, the present data showed that auraptene might be responsible for its cytotoxic and anticancer properties in U87 cells. As shown in Figure 7(Fig. 7), we have demonstrated the proposed mechanisms of auraptene in the U87 GBM cell line. 

## Conclusions

In summary, the outcomes of the current study provide the first evidence that auraptene-induced ROS generation mediates cytotoxicity and disrupts apoptosis via Bax/Bcl-2 regulation and Cyclin D1, p21, and CXCL3 genes modulation in GBM cells. Due to its relative non-lethal nature and its ability to induce apoptosis of U87, auraptene could be a promising novel natural candidate for the therapy of GBM patients, after further mechanistic studies.

## Declaration of interest

The authors declare that they have no competing interests.

## Acknowledgements

This work was partly supported by Mashhad University of Medical Sciences (Grant No. 951265) and Bu Ali Research Institute, Mashhad, Khorasan Razavi, Iran for their technical assistance. 

The authors would like to honor *Dr. Sima Khosravi*, a kind physician and a great mother to the first author (ARA), who lost her battle with GBM disease in the fall of 2016.

## Figures and Tables

**Table 1:** The sequence of primers in the present study

**Figure 1:** Chemical structure of auraptene

**Figure 2:** (A) Effects of auraptene on ROS levels in U87 cells. Auraptene decreased ROS levels in the early hours (2 and 6 hours) but enhances ROS generation in the 24 hours after treatment. Cells were treated for 2, 6, 8, and 24 hours at auraptene concentrations of 50, 100, and 200 μg/mL, and the ROS was measured by a fluorimeter (Epoch, BioTek^®^ instruments, Inc, USA). In the TBHP positive control (150 μM) sample, the fluorescence intensity increased significantly compared to the control group. Also, N-acetyl-cysteine (NAC, five mM) decreased the auraptene-induced ROS production at 8 and 24 hours after treatment, significantly. Each column represents the mean±standard error in the samples. (^#^p<0.05, ^##^p<0.01 and ^###^P<0.001 compared with control) (n=4). (B) NAC (five mM) plus auraptene increased the cell viability at 8 (concentration of 50 μg/mL) and 24 (50, 100 and 200 μg/mL) hours after treatment compared with each other group. Each column shows the mean±standard error in the samples. (^###^P<0.001 and ^#^p<0.05 compared with the control group, **p<0.01 and *p<0.05 compared with each other group in the same concentration) (n=4)

**Figure 3:** (A) The measurement of apoptotic and necrotic cells was performed by the annexin V-FITC/PI staining assay 24 hours after treatment by auraptene (100 and 400 μg/mL). Auraptene induced apoptosis concentration-dependently 24 hours after treatment compared to the control group. FL2-H and FL1-H are PI and annexin V-FITC, respectively. The annexin V-FITC conjugated protein was bound to the phosphatidyl serine-expressing cell surface, which is an early apoptosis marker. The cells were stained with PI, a non-penetrating color to the DNA, indicating necrotic cells. The cells stained with PI and annexin V-FITC represent the endpoints of apoptosis and the initial phase of necrosis. The percentages of viable, early/late apoptotic, and necrotic cells in the treated samples compared to the control group, 24 hours after treatment by auraptene (Q1: annexin V−/PI +, necrotic cells; Q2: annexin V+ /PI +, late apoptotic cells; Q3: annexin V+ /PI −, early apoptotic cells; Q4: viable cells). Tests were repeated in triplicate. (B) and (C) show the percentage of apoptosis process in each phase and the apoptotic and necrotic index in the treated samples as compared with the control group, 24 hours after treatment, respectively. Each column represents the mean ± standard error in the samples. ***P<0.001 as compared with the control group (n=5)

**Figure 4:** (A) The measurement of apoptotic and necrotic cells was performed by the annexin V-FITC/PI double-staining assay 48 hours after treatment by auraptene (100 and 400 μg/mL). Auraptene induced apoptosis concentration-dependently manner 24 hours after treatment compared to the control group. FL2-H and FL1-H are PI and annexin V-FITC, respectively. The annexin V-FITC conjugated protein was bound to the phosphatidyl serine-expressing cell surface, which is an early apoptosis marker. The cells were stained with PI, a non-penetrating color to the DNA, indicating necrotic cells. The cells stained with PI and annexin V-FITC represent the endpoints of apoptosis and the initial phase of necrosis. The percentages of viable, early/late apoptotic, and necrotic cells in the treated samples compared to the control group, 48 hours after treatment by auraptene (Q1: annexin V−/PI +, necrotic cells; Q2: annexin V+ /PI +, late apoptotic cells; Q3: annexin V+ /PI −, early apoptotic cells; Q4: viable cells). Tests were repeated in triplicate. (B) and (C) show the percentage of apoptosis process in each phase and the apoptotic and necrotic index in the treated samples as compared with the control group, 48 hours after treatment, respectively. Each column represents the mean±standard error in the samples. *** P<0.001 as compared with the control group (n=5)

**Figure 5:** The U87 cells were treated with the indicated concentrations of auraptene for 24 hours. Total RNA was isolated, and RT-PCR analyzed mRNA expression. The relative genes expression levels of p21 (A), Cyclin D1 (B), and CXCL3 (C) were determined by densitometer analysis. The y-axis indicates the fold-change. Results were normalized to levels of GAPDH in the samples. *P<0.05, **P<0.01 and ***P < 0.001 compared to the control group

**Figure 6:** (A) Auraptene suppresses Bcl-2 protein expression in U87 cells and up-regulates Bax protein level. U87 cells were treated with 100 and 400 μg/mL of auraptene for 24 hours. The total protein levels of Bax and Bcl-2 are assessed by Western blotting. The relative density of Bax and Bcl-2 are determined by densitometry of the blots using Image J 1.52a software and were compared to the β-actin protein. **p<0.01 and ***P<0.001 compared to the control group. (B) Auraptene increased the Bax/Bcl-2 protein ratio after 24 hours' treatment, significantly. *p<0.05 and ***P<0.001 compared to the control group

**Figure 7:** The proposed model of molecular signaling pathways from U87 cells following exposure to auraptene
